# Cilengitide Inhibits Neovascularization in a Rabbit Abdominal Aortic Plaque Model by Impairing the VEGF Signaling

**DOI:** 10.1155/2021/5954757

**Published:** 2021-11-30

**Authors:** Fawang Zhu, Shuai Yuan, Jing Li, Yun Mou, Zhiqiang Hu, Xiuqin Wang, Xiaotong Sun, Jie Ding, Zhelan Zheng

**Affiliations:** ^1^Department of Echocardiography and Vascular Ultrasound Center, The First Affiliated Hospital, Zhejiang University School of Medicine, 79 Qingchun Road, Hangzhou, Zhejiang Province 310003, China; ^2^Zhejiang University School of Medicine, 866 Yuhangtang Road, Hangzhou, Zhejiang Province 310023, China

## Abstract

**Background:**

Cilengitide is a selective *α*_v_*β*_3_ and *α*_v_*β*_5_ integrin inhibitor. We sought to investigate the effect of cilengitide on the neovascularization of abdominal aortic plaques in rabbits and explore its underlying antiangiogenic mechanism on human umbilical vein endothelial cells (HUVECs).

**Materials and Methods:**

For the *in vivo* experiment, the abdominal aortic plaque model of rabbits was established and injected with different doses of cilengitide or saline for 14 consecutive days. Conventional ultrasound (CUS) and contrast-enhanced ultrasound (CEUS) were applied to measure the vascular structure and blood flow parameters. CD31 immunofluorescence staining was performed for examining neovascularization. Relative expressions of vascular endothelial growth factor (VEGF) and integrin of the plaque were determined. For *in vitro* experiments, HUVECs were tested for proliferation, migration, apoptosis, and tube formation in the presence of different doses of cilengitide. Relative expressions of VEGF, integrin, and Ras/ERK/AKT signaling pathways were determined for the exploration of underlying mechanism.

**Results:**

CEUS showed modestly increased size and eccentricity index (EI) of plaques in the control group. Different degrees of reduced size and EI of plaques were observed in two cilengitide treatment groups. The expressions of VEGF and integrin in the plaque were inhibited after 14 days of cilengitide treatment. The neovascularization and apoptosis of the abdominal aorta were also significantly alleviated by cilengitide treatment. For *in vitro* experiments, cilengitide treatment was found to inhibit the proliferation, migration, and tube formation of HUVECs. However, cilengitide did not induce the apoptosis of HUVECs. A higher dose of cilengitide inhibited the mRNA expression of VEGF-A, *β*_3_, and *β*_5_, but not *α*_V_. Lastly, cilengitide treatment significantly inhibited the Ras/ERK/AKT pathway in the HUVECs*. Conclusions*. This study showed that cilengitide effectively inhibited the growth of plaque size by inhibiting the angiogenesis of the abdominal aortic plaques and blocking the VEGF-mediated angiogenic effect on HUVECs.

## 1. Introduction

Stabilizing vulnerable plaque to prevent the occurrence and development of acute cardiovascular and cerebrovascular events is an important goal for the medical community [1]. Vulnerable plaque is prone to rupture and thrombosis, which blocks the arterial blood supply resulting in cardiocerebrovascular diseases and death. Neovascularization of plaque in arteries is an important factor leading to the rupture of vulnerable plaque [2, 3]. At present, the clinical treatment of plaque is limited, and stabilization with statins is far from ideal [4–6].

Angiogenesis is the formation of new capillaries from preexisting blood vessels. It is regulated by proangiogenic and antiangiogenic factors. Among the proangiogenic factors, vascular endothelial growth factor (VEGF) is the most widely understood mediator in angiogenesis [2]. VEGF plays a vital role in pathological angiogenesis, promoting the development of pathological processes, including tumor growth and metastasis, inflammation, and myocardial ischemia [6–8]. Previous studies have also emphasized that proangiogenic therapy enhances atherosclerosis, while antiangiogenic therapy reduces atherosclerotic complications. Hence, antiangiogenic therapy may be a promising strategy for treating atherosclerosis [9].

Integrin-mediated signaling is essential for stabilizing cell adhesion and promoting cell migration, proliferation, and survival [3, 10]. Integrin adhesion receptor-mediated endothelial cell-matrix interaction plays a crucial role in vascular development, angiogenesis, and vascular homeostasis. Many studies have indicated that integrin inhibitors effectively inhibit neovascularization in tumors, thereby inhibiting tumor growth [3, 11, 12].

Cilengitide (EMD121974) is a cyclic arginine-glycine-aspartate- (RGD-) derived peptide that has a high affinity for integrin *α*_v_*β*_3_ and inhibits integrin *α*_v_*β*_3_ and *α*_v_*β*_5_ functions. Previous studies have confirmed that cilengitide can inhibit angiogenesis and migration in various tumors and promote the apoptosis of vascular endothelial cells, thus inhibiting tumor development [11]. Although phase 3 trials of cilengitide as an antitumor therapy failed to show improved outcomes, the effect of cilengitide on normal vascular endothelial cells has not been clarified [12]. The purpose of this study was to explore the stabilizing and inhibitory effects of the integrin inhibitor cilengitide on neovascularization in plaques and determine the underlying antiangiogenic mechanism on human umbilical vein endothelial cells (HUVECs).

## 2. Materials and Methods

### 2.1. Experimental Animals

Twelve male New Zealand white rabbits weighing 2.6-3.1 kg (2.811 ± 0.142 kg) were provided by the Zhejiang University Experimental Animal Center (animal permit approval number: SCXK (Zhe) 2017-0004). The experimental animal protocol was approved by the Institutional Animal Care and Use Committee of Zhejiang University (approval number: ZJU20190070). The disposal of euthanized animals during the experiments conformed to the Laboratory Animal-Guideline for ethical review of animal welfare (approval number: GB/T 35892-2018) and was approved by the Animal Experimentation Ethics Committee of Zhejiang University. The high-fat feed consisted of 10% lard + 3% cholesterol + 87% essential ingredients at ordinary levels and was bought from Beijing Keao Xieli Feed Co., Ltd. (Beijing, China) (Approval number: SCXK (Jing) 2019-0003).

### 2.2. Establishment of the Aortic Plaque Model

The rabbits were anesthetized with 3% pentobarbital sodium (30 mg/kg) intravenously. The right femoral artery was then freed under sterile operating conditions after local shaving and disinfection. Following a successful puncture of the femoral artery with a 24-gauge indwelling needle, the Choice PT guidewire was fed to the thoracic aorta using a retrograde approach. A 3.5 mm × 15.0 mm balloon catheter was introduced into the descending aorta about 20 cm along the guidewire. After filling the balloon to 8 standard atmospheric pressure, it was pulled back to the iliac artery at a constant speed for about 5 seconds each time. The abdominal intima was injured five times. The right femoral artery was ligated, and the wound was sutured. After the operation, an intramuscular injection of 400,000 IU/day penicillin was administered for three consecutive days to prevent infection. The rabbits were returned to their housing room and fed with a high-fat feed at 200 g/day.

### 2.3. Performance of CUS and CEUS

After continuous feeding for 8-10 weeks, the abdominal aortas of model animals were examined with conventional ultrasound (CUS) and contrast-enhanced ultrasound (CEUS) before cilengitide treatments. Local intima-media thickness (IMT) of ≥0.5 mm containing contrast medium was used to indicate that the abdominal aortic plaque model had been established. The inner diameter, peak systolic velocity (PSV), and resistance index (RI) of the abdominal aorta were routinely measured. Simultaneously, the number, position, and size of each plaque, as well as the vascular remodeling index (VRI) and the plaque eccentricity index (EI), were measured and calculated by CEUS. These parameters were then evaluated again after the cilengitide treatment for comparison. The amount of contrast agent in the plaque was evaluated from the number of points reflecting the degree of blood perfusion in the plaque. All ultrasound examinations were performed as blind procedures by an individual ultrasound expert.

VRI was calculated as VRI = total vessel area (TVA) at the plaque/TVA of the plaque reference sites [13]. The TVA is defined as the cross-sectional area of the blood vessel surrounded by the mid-outer membrane junction of the arterial wall. The TVA of the plaque reference vessel sites is defined as the average TVA, both 1 cm proximal and 1 cm distal to the plaque. Plaque EI was calculated as EI = (thickest IMT − thinnest IMT)/thickest IMT [14]. Schematics of the TVA and the EI are shown in Figures 1(a) and 1(b), respectively.

### 2.4. Cilengitide Treatment

Twelve rabbits with abdominal aortic plaques, confirmed by CUS, were randomly divided into three groups (*n* = 4 each): T0, T1, and T2 groups. Cilengitide was purchased from MedChemExpress (MCE, Princeton, NJ, USA) and was dissolved in dimethyl sulfoxide (DMSO) with a concentration of 100 mg/mL for storage. Before injecting, cilengitide was diluted into a final concentration of 100 *μ*g/mL with saline and administered once daily by intravenous injection in the T2 (200 *μ*g/day) and T1 (100 *μ*g/day) groups. The T0 group was injected with saline using the same volume of cilengitide administered to the T1 group. All groups were treated continuously for 14 days. During the treatment, one accidental death occurred in each of the T1 and T0 groups. On the 15th day, the inner diameter, IMT, PSV, RI of the abdominal aorta, plaque size, and EI at the original mark were measured and recorded by CUS. If new plaque formation was found, the location, size, and echo characteristics of the new plaque were measured and recorded. The degree of contrast agent perfusion was simultaneously analyzed by CEUS.

### 2.5. Histological Analysis

After cilengitide treatment for 14 consecutive days, the degree of plaque in the abdominal aorta was evaluated by CUS and CEUS. Each plaque's location was recorded by calculating its distance to the right kidney artery during the ultrasound. The rabbits were anesthetized by 3% pentobarbital based on body weight (3.0 mL/kg) and sacrificed. Their abdominal aortas were separated. Each aorta specimen was cut to a length of 8 cm according to the ultrasound-labeled plaque position. The plaques were then precisely located by calculating their distances from the right kidney. Each plaque was cut into two halves, one for the histological analysis and the other for the molecular experiment. The former ones of the aorta were fixed in 4% paraformaldehyde for 24 h and embedded in paraffin. Then the samples were serially sectioned. The sections were performed with the haematoxylin-eosin (H&E) staining, Movat-Russell modified pentachrome (Movat) staining, CD31-positive staining (Abcam, USA), and terminal deoxynucleotidyl transferase dUTP nick end labeling (TUNEL) staining. The Movat staining was conducted according to the protocol of the commercial kit (Solarbio, Beijing, China). The TUNEL staining was performed following the instruction of the In Situ Cell Death Detection Kit (Roche, USA). The points merged by green (TUNEL) and blue (DAPI) were considered the TUNEL-positive cell. The ratios of TUNEL-positive cell and DAPI-positive cell were calculated as the TUNEL-positive cell percentage.

### 2.6. Tissue Extraction and Protein Level Detection

The aortas containing the plaques were washed with cold normal saline and quickly removed. A part of the aorta was stored in the freezer at -80°C for uniform testing of western blotting and reverse transcription-quantitative polymerase chain reaction (RT-qPCR), and the rest was used for the ELISA assay. The mRNA and protein levels of VEGF-A were determined by RT-qPCR and western blotting, respectively. Meanwhile, the absolute protein contents of VEGF-A and VEGFR2 were examined by the ELISA kit (Thermo Fisher Scientific, USA) according to the protocol of the manufacturer.

### 2.7. Cell Culture

HUVECs were purchased from American Type Culture Collection (ATCC, Manassas, VA, USA). We cultivated the cell in low-glucose Dulbecco's modified Eagle medium (DMEM; Hyclone, Logan, UT, USA) supplemented with 10% fetal bovine serum (FBS; Biological Industry, Israel), 100 U/mL penicillin, and 100 ng/mL streptomycin (Invitrogen, Carlsbad, CA, USA). Cells were incubated at 37°C in an atmosphere with 5% CO_2_. Cells between passages 5-15 were then utilized. Before plating cells, the cell plates were added with 2 *μ*g/mL vitronectin (Solarbio, Beijing, China) at 4°C overnight in cell experiments except for tube formation assay. For proliferation, apoptosis, and migration assays, cells were cultured in DMEM alone overnight for starvation. Cells treated with 0 *μ*M cilengitide were used as a control group and received DMSO in the same volume as the other groups that received cilengitide.

### 2.8. Proliferation Assay

Cells were seeded in duplicate in 96-well plates at a density of 8 × 10^3^ and then cultured for 24 hours without or with cilengitide at different concentrations. Cell viability was monitored by a Cell Counting Kit-8 (CCK-8) (Dojindo, Kumamoto, Japan). Briefly, CCK-8 reagents (10 *μ*L) were added to each well and incubated for 1 hour at 37°C. The absorbance at 450 nm was measured by a microplate reader to assess the number of viable cells.

### 2.9. Migration Assay

HUVEC migration was measured by a wound-healing migration assay. Cells were seeded in a 6-well tissue culture plate at a density of 3 × 10^4^ and cultured at 37°C for 24 hours. Scratch wounds were created by scraping the cell monolayer with a sterile 10 *μ*L pipette tip. HUVECs were starved by culturing in DMEM without FBS overnight, then treated with cilengitide at different concentrations at 37°C for 24 hours. Untreated cells were used as controls. The migrated cells were imaged in five randomly selected fields of view with a phase-contrast microscope (Nikon, Tokyo, Japan). The percentage of migration was analyzed by the ImageJ software (National Institutes of Health, Bethesda, MD, USA).

### 2.10. Flow Cytometry Analysis of Apoptosis

Annexin V-fluorescein isothiocyanate (FITC)/propidium iodide (PI) double staining was used to detect cell apoptosis. HUVECs were plated in 6-well tissue culture plates at a density of 3 × 10^4^ per well. After exposure to 0-10 *μ*M cilengitide, the cells were collected and washed twice with phosphate-buffered saline (PBS), then resuspended in binding buffer at 1 × 10^6^ cells/mL. This suspension was incubated in 5 *μ*L Annexin V-FITC and PI solutions for 15 minutes in the dark at room temperature. Flow cytometric analysis of apoptosis was performed within 1 hour.

### 2.11. Endothelial Cell Tube Formation Assay

HUVECs (2 × 10^4^ cells/well) together with different concentrations (0-10 *μ*M) of cilengitide were plated on polymerized Matrigel (growth factor reduced) (Solarbio, Beijing, China) in 96-well plates. Untreated cells were used as controls. After 8 hours of incubation at 37°C in a cell culture incubator, tube-like structure formation was imaged using an inverted microscope (Nikon, Tokyo, Japan). The length of tubes, tube areas, and the number of capillary-like structures were quantified from representative fields using the ImageJ software.

### 2.12. Reverse Transcription-Quantitative Polymerase Chain Reaction (RT-qPCR)

Using the TRIzol reagent (Invitrogen), total RNA was isolated from the arterial tissue or cell samples as previously described. The mRNA was converted into cDNA and performed with quantitative PCR using SYBR® Premix Ex Taq™ II (Takara) by the 7500 Fast Real-Time PCR System (Applied Biosystems, Foster, CA, USA). *β*-Actin and GAPDH expression were used for normalization in *in vivo* and *in vitro* experiments, respectively. PCR primers were synthesized at Sangon Biotech (Shanghai, China) (see Table 1). PCR products were quantified using the 2^−*ΔΔ*Ct^ method.

### 2.13. Western Blotting

Frozen abdominal aorta specimens were lysed by RIPA containing phenylmethylsulfonyl fluoride (PMSF) and homogenized with a homogenizer. Then, the lysis buffer was separated by centrifugation at 14,000 g/min for 5 minutes at 4°C, and the supernatant was taken for western blotting. Similarly, the cell samples were lysed by RIPA containing PMSF and collected for detection of the protein expressions. Total protein concentrations were confirmed by a BCA protein assay kit (Thermo Scientific, Waltham, MA, USA). Protein samples, 20-50 *μ*g of each, were separated by sodium dodecyl sulfate-polyacrylamide gel electrophoresis (SDS-PAGE) and transferred to polyvinylidene fluoride (PVDF) membranes. After blocking with 5% bovine serum albumin in Tris-buffered saline containing 0.1% Tween 20 (TBST) for 1 hour at room temperature, the membranes were incubated at 4°C with primary antibodies overnight as follows: VEGF-A (1 : 1000, ab1316, Abcam), MCP-1 (1 : 1000, 66272-1-Ig, ProteinTech), MMP-2 (1 : 1000, ab97779, Abcam), MMP-9 (1 : 1000, ab58803, Abcam), p-ERK (1 : 1000, #9101, CST), ERK (1 : 1000, #4695, CST), p-AKT (1 : 1000, #4060, CST), AKT (1 : 1000, #4691 CST), Ras (1 : 1000, ab108602, Abcam), and *β*-actin (1 : 1000, ab8227, Abcam). The membranes were then washed with TBST three times and incubated with the secondary antibody (1 : 2000, SA00001-1, and SA00001-2, ProteinTech) at room temperature for 1 hour. After washing three times with TBST, the membranes were visualized with an enhanced chemiluminescence detection kit (Bio-Rad, Hercules, CA, USA). Antibodies against GAPDH, ERK, and AKT were used as internal references. ImageJ was used to analyze the relative quantity of each protein.

### 2.14. Statistical Analysis

Experiments were repeated at least three times. All experimental data are presented as the mean ± standard error of the mean (SEM). A two-tail unpaired *t*-test was used to compare differences between two groups, and one-way ANOVA was applied for the comparison among three or more groups. The control group was set up as 1 for each independent experiment; thus, the SEM for controls was zero. All statistical analyses were performed by GraphPad Prism 8.0. Differences with a *p* value < 0.05 were considered statistically significant.

## 3. Results

### 3.1. Cilengitide Inhibited the Growth of Plaques in the Abdominal Aorta

One rabbit died unexpectedly in groups of T1 and T0, while the rest model animals completed the experiment. We totally detected three, five, and seven plaques by CUS and CEUS before cilengitide treatment among the model animals in T0, T1, and T2 groups, respectively. It indicated the successful establishment of the abdominal aortic plaque model. Then, the changes of each plaque were recorded before and after the cilengitide treatment. Both CUS and CEUS examinations provided adequate images of abdominal aortic plaques in model animals. However, the CEUS showed the plaque boundary more clearly (see Figure 2).

Evaluated by CUS, we found that there were no statistically significant differences in basic parameters of the abdominal aorta (inner diameter, IMT, and PSV), RI, and VRI among the three groups before or after cilengitide treatments (*p* value > 0.05 for all comparisons, Table 2). Besides, the plaque size and EI among the three groups at baseline also showed no significant differences before cilengitide treatment (*p* value > 0.05 for all comparisons, Table 3). After cilengitide treatment, CUS examination showed shrinking of the plaques and a slight decrease of EI in all three groups, while those changes showed no significant differences among the three groups (Table 4). In comparison, CEUS examination indicated a slight increase in the abdominal aortic plaque size and EI in the T0 group, which decreased in the T1 and T2 groups. The changes of anteroposterior diameter (AD) and EI in the T1 group showed significant differences from those in the T0 group. Besides, the longitudinal diameter (LD), AD, and EI of the plaques in the T2 group were also significantly different from those in the T0 group (Table 4). The representative image for CUS and CEUS examination in the T2 groups is shown in Figure 3. It showed shrinking of the plaque after the cilengitide treatment by both CUS and CEUS examination. These results indicated that the integrin *α*_v_*β*_3_ inhibitor cilengitide could effectively inhibit the growth of abdominal aortic plaques in model rabbits. It appeared that the higher-dose treatment (200 *μ*g/day) might have been more effective.

### 3.2. Cilengitide Inhibited the Growth of Plaques, Neovascularization, and Apoptosis in the Abdominal Aorta

Evaluated by H&E and Movat staining, cilengitide treatment significantly inhibited the growth of the plaques since the plaques in the T1 and T2 groups were less, and the sizes of the plaque were smaller compared with that in the T0 group (Figure 4). To evaluate the effect of cilengitide on neovascularization, we conducted the CD31 staining to observe the microvessels within the plaque. The abdominal aorta in the T0 group showed numerous CD31-positive microvessels in the plaque, while such microvessels were significantly decreased after cilengitide treatments in the T1 and T2 groups (Figure 5). Besides, we performed the TUNEL staining to show the apoptosis of the abdominal aorta. The T1 and T2 groups showed fewer TUNEL-positive cells than the T0 group, and the differences were both significant (Figure 6). These results indicated that cilengitide treatment could effectively inhibit the growth of the plaques and apoptosis of the abdominal aorta in the model rabbits.

### 3.3. Cilengitide Decreased the VEGF, MMP-2, MMP-9, and MCP-1 Expression in the Abdominal Aortic Plaques

To provide evidence that cilengitide has a protective effect on neovascularization in abdominal aortic plaques, we examined the expression of VEGF-A and VEGFR-2 in abdominal aortic tissue in the three groups. We set the samples from random normal blood vessels taken >3 cm away from the plaque area as the control group. The expressions of VEGF-A and VEGFR-2 were significantly increased in the T0 group compared with the control group (Figures 7(a)–7(e)). Treatment with cilengitide at 100 *μ*g or 200 *μ*g per day (T1 and T2 groups) significantly reduced these elevated expression levels. Also, we confirmed the effect of cilengitide on integrin expression. The relative mRNA expressions of *α*_v_, *β*_3_, and *β*_5_ were all inhibited in the T1 and T2 groups compared with those in the T0 group (Figures 7(f)–7(h)). These results demonstrated that cilengitide could effectively inhibit VEGF expression in abdominal aortic plaques and plaques' growth in model rabbits. We then investigated the role of cilengitide on plaque stability, indicated by the relative expression of matrix metalloproteinases (MMPs). Secreted by macrophages, MMP-2 and MMP-9 also play critical roles in intraplaque angiogenesis. MCP-1 is expressed by inflammatory cells and a potent stimulus of monocyte recruitment. Consistently, cilengitide treatment effectively inhibited the increased protein expression of MM9-2, MMP-9, and MCP-1 in the plaques (Figures 7(i)–7(l)).

### 3.4. Cilengitide Attenuated Cell Proliferation, Migration, Invasion, and Tube Formation but Not Affected the Apoptosis of HUVECs

To evaluate the inhibitory effect of cilengitide in angiogenesis, HUVECs were treated with different doses of cilengitide. The viability of HUVECs reflected by the CCK-8 assay was significantly reduced after 1 *μ*M or 10 *μ*M of cilengitide treatment (Figure 8(a)). The inhibitory effect of cell proliferation was enhanced as the cilengitide concentration was increased. Meanwhile, wound-healing assays showed that the cell migration capacity of HUVECs was significantly inhibited by treatment with 10 *μ*M cilengitide for 6 to 24 hours. However, there were no significant differences between cells treated with no cilengitide group and lower concentrations groups (0.1 *μ*M and 1 *μ*M; Figures 8(b) and 8(c)). Interestingly, flow cytometry analysis revealed that no significant increase of apoptosis was observed for HUVECs when treated with 0.1-10 *μ*M cilengitide for 24 hours (Figures 8(d) and 8(e)). The tube formation experiment was then produced to investigate the angiogenic ability of HUVEC after cilengitide treatment. The tube network formation on the Matrigel matrix showed that a lower dose of cilengitide (0.1 *μ*M) could significantly reduce the length of the tube. Higher doses of cilengitide (1 *μ*M and 10 *μ*M) also inhibited the length of the tube, tube areas, and the number of capillary-like structures (Figures 8(f)–8(i)). These findings demonstrated that cilengitide could influence the proliferation, migration, and tube formation of HUVECs but did not induce increased apoptosis.

### 3.5. Cilengitide Reduced mRNA Expression of VEGF-A and Integrins of HUVECs

We explored the underlying mechanism of the cilengitide on the HUVECs. The mRNA expressions of VEGF-A and integrins were detected. Compared with the no cilengitide treatment group, the mRNA expression levels of VEGF-A, integrins *β*_3_, and integrins *β*_5_ under 10 *μ*M cilengitide were significantly decreased (Figure 9). In contrast, the mRNA expression of *α*_V_ was not significantly changed by any doses of cilengitide.

### 3.6. Cilengitide Reduced Protein Expression of VEGF-A and Inhibited VEGF Downstream Pathways of HUVECs

Lastly, we explored the protein expression of VEGF-A, Ras, p-ERK/ERK, and p-AKT/AKT in HUVECs by the cilengitide treatment. Cilengitide treatment at 1 *μ*M and 10 *μ*M for 1 hour led to significant decreases in the protein expression levels of VEGF-A and Ras (Figure 10). Meanwhile, the protein expression ratios of p-ERK/ERK and p-AKT/AKT were also decreased. However, 0.1 *μ*M cilengitide treatment has no apparent inhibitory effect on these protein expressions. The main finding of cilengitide on the HUVECs was summarized in Figure 11.

## 4. Discussion

About 75% of acute coronary syndromes and most symptomatic carotid artery diseases are caused by rupture of vulnerable plaque [15]. Neovascularization and bleeding within the plaque are essential factors in the formation of vulnerable plaque [16]. There is increasing histopathologic evidence that vulnerable plaque contains more new blood vessels than stable plaque [17]. Such neovascularization in plaque is closely related to its rapid progress and transition to vulnerable plaque, with intimal neovascularization being a characteristic manifestation of most atherosclerotic diseases [18].

Integrin *α*_v_*β*_3_ has a critical regulatory role in neovascularization [19, 20]. Antibodies and small inhibitors of integrin (such as RGD cyclic peptides) have been previously used to successfully prevent angiogenesis by inhibiting the binding of ligands to integrin and subsequently blocking the adhesion function of integrin *α*_v_*β*_3_, thereby decreasing neovascularization and VEGF-A content [20]. The growth, migration, and vascular proliferation of solid tumors were also inhibited by antagonists of integrin *α*_v_*β*_3_ in animal models [21]. The integrin inhibitor cilengitide can selectively inhibit *α*_v_*β*_3_ expression at an IC50 ranging from 3 to 40 nmol/L, which is about ten times more selective than platelet membrane glycoprotein IIb/IIIa [22]. The expression of integrin *α*_v_*β*_3_ is low in mature vascular endothelial cells and most normal tissues and organs in healthy people. Increased integrin *α*_v_*β*_3_ expression and neovascularization are essential features in the development of all vulnerable plaques, suggesting a particular specificity of integrin *α*_v_*β*_3_ for this process [23]. Thus, integrin inhibitor cilengitide is a theoretically feasible and effective treatment for atherosclerotic plaques.

In this study, we first established the abdominal aortic plaque model in rabbits and detected the plaque sizes using CUS and CEUS simultaneously. For the model group, a slight decrease of plaques was observed by CUS. However, the images detected by CUS were insufficient to provide detail of plaques. Previous studies have proved the great advantages of CEUS in the imaging of neovascularization within atherosclerotic plaques *in vivo* compared with CUS [24, 25]. In this study, the CEUS experiments showed that the contrast agent was visible in the abdominal aortic plaques, indicating neovascularization in the plaques. So the plaque sizes were shown more clearly and precisely by CEUS. It showed that the plaques in the T0 group were increased. The VEGF-A and VEGFR-2 expressions increased in plaques, which might activate the integrin *α*_v_*β*_3_ [26, 27]. After 14 consecutive days of cilengitide treatment, cilengitide appeared to achieve stability and inhibit the growth of plaques and even reverse reconstruction. The ultrasound examination showed that plaques in the abdominal aorta became smaller, and the plaque EI decreased in the cilengitide treatment groups. The higher-dose treatment group showed more apparent inhibition of abdominal aortic plaque progression. The VEGF-A and VEGFR-2 expressions were also reduced after cilengitide treatment. It was possible that the inhibition of integrin *α*_v_*β*_3_ by cilengitide led to decreased VEGF-A expression, thereby inhibiting neovascularization in the plaque.

The plaque EI is a direct and early reflection of vascular blood flow that can also reflect vascular remodeling to some extent [14]. Our experiments showed a statistically significant decrease in EI after cilengitide treatment, indicating that the local internal diameter and blood flow of the vessel increased. However, the VRI did not change significantly after the cilengitide treatment. Atherosclerotic vascular remodeling includes arterial wall shrinkage (negative remodeling) with a VRI < 0.95 and arterial compensated expansion (positive remodeling) with a VRI ≥ 1.05 [28]. In our study, the VRIs in this study of all groups were between 0.95 and 1.05, indicating no remodeling of the abdominal aorta. One possible explanation for this result is that the relatively small size of the experimental plaques was insufficient to cause blood flow changes, compensatory expansion, or contraction of blood vessels.

To determine the potential mechanism, we detected several indicators of angiogenesis and inflammation in the plaque of the abdominal aorta. Firstly, we confirmed that the contents of VEGF-A and VEGF-R2 were enhanced in the T0 group. Consecutive injection of cilengitide could inhibit these protein contents, as well as the mRNA expression of integrin. Furthermore, a previous study [29] has found that the MMP-2 and MMP-9, two important proangiogenic mediators within the plaque, were evaluated in the plaque and promoted plaque stability. Inhibition of MMPs was considered an effective therapeutic target for preventing the rupture of plaque. Meanwhile, another critical proinflammatory indicator, MCP-1, plays an essential role in responding to inflammation. It can recruit monocytes and promote inflammation within the plaque, further inducing the instability of plaques. Our results showed that cilengitide also has a suppressive effect on the MMP-2, MMP-9, and MCP-1 expression, which might be the potential mechanism of cilengitide in stabilizing the plaque.

Vascular endothelial cells (ECs) acted as sensors and effectors of the vessels that secreted various vasoactive substances against multiple stimulations. The changes regulated by ECs could affect vascular structure and function [30]. So we also performed *in vitro* study to further explore the effect of cilengitide on the HUVECs. We found that cilengitide inhibited the proliferation, migration, and tube formation of HUVECs, similar to those findings in the tumor cells [31, 32]. However, there was no significant effect on the apoptosis of HUVECs. These findings suggested that cilengitide might inhibit the angiogenesis of normal endothelial cells without causing cell death, which showed a preferential application for cilengitide.

VEGF is one of the major angiogenic growth factors that regulate angiogenesis. The VEGF gene family includes VEGF-A, VEGF-B, VEGF-C, VEGF-D, VEGF-E, and PGF. Of these, VEGF-A plays a significant role and is highly expressed in atherosclerotic plaques. Recognized by VEGF receptors, primarily VEGFR-2, VEGF-A promotes endothelial cell proliferation, differentiation, and migration. Besides, it participates in neovascularization through different signaling pathways, such as Ras, ERK, and AKT pathways [33, 34]. In this study, we observed an inhibitory effect of cilengitide on the VEGF-A and VEGFR-2 expression in the vulnerable plaques and the VEGF-A expression at both mRNA and protein levels in HUVECs, thus potentially inhibiting the growth of neovascularization in the plaque model.

We also showed that cilengitide downregulated the expression of integrins *β*_3_ and *β*_5_, but not *α*_V_. The mechanism of this regulation of integrin expression needs further investigation. Besides, we found that cilengitide inhibited the PI3K/AKT and Ras/MAPK pathways, which were classical pathways that regulated cell proliferation, differentiation, and survival. Collectively, integrin *α*_v_*β*_3_ is not only a potential target molecule for tumor diagnosis and treatment but is also a specific target for molecular imaging and treatment of vulnerable plaques [35, 36]. These results may provide an important experimental and theoretical basis for new approaches to the clinical prevention and treatment of atherosclerotic plaque.

There are some limitations to this study. First, the number of rabbits was limited, and our use of only two doses groups was insufficient to determine the optimal cilengitide concentration to inhibit plaque growth and reverse remodeling. Second, we just tested a two-week treatment duration, which did not provide information on long-term efficacy. Third, we did not test whether the rabbit's abdominal aortic plaques would stop growing or even become smaller after the high-fat diet is stopped, with or without drug treatment. Besides, the inhibitory role of cilengitide on the Ras/ERK/AKT signaling pathway was only an observational result. Direction evidence was not provided between the reduced VEGF expression and this signaling pathway. Finally, the contrast agents used in this study, micron-level microbubbles, were limited for visualizing contrast in plaque. It is hoped that developing smaller (e.g., nanolevel) contrast agent microbubbles might allow more contrast agents to enter into the new blood vessels resulting from angiogenesis in plaque.

## 5. Conclusions

Cilengitide effectively inhibited neovascularization and plaque growth in the abdominal aortic plaque models in a rabbit model by reducing the expression of VEGF. Cilengitide also inhibited normal endothelial cell proliferation, migration, and tube formation without leading to cell death. One mechanism for the inhibitory effect of cilengitide on HUVECs is the regulation of VEGF expression. Further studies are needed to reveal the mechanism of cilengitide regulation of integrin gene expression.

## Figures and Tables

**Figure 1:** Schematic diagram of the total vessel area (TVA) and the eccentricity index (EI). (a) The grey ellipse in the lower two vessels represents TVA. (b) The components and calculation formula for EI.

**Figure 2:** Visualization of representative abdominal aortic plaques and contrast agent perfusion in different imaging modes in the T2 group. (a) Plaque on CUS. (b) The boundary of the plaque is shown more distinctly on CEUS. (c) The clear appearance of contrast agent microbubbles in the plaque.

**Figure 3:** Ultrasound images of a representative plaque in the T2 group in different imaging modes and at different periods. (a) Pretreatment on CUS. (b) Pretreatment on CEUS. (c) Posttreatment on CUS. (d) Posttreatment on CEUS.

**Figure 4:** Representative image for H&E and Movat staining. (a) The representative image for H&E staining. (b) The representative image for Movat staining.

**Figure 5:** Cilengitide inhibits neovascularization within the plaque of the abdominal aorta. (a) The representative image for CD31-positive staining. The white arrow indicates the CD31-positive microvessels in the plaque. Scale bar, 100 *μ*m. (b) Quantitative results of CD31-positive cells. *n* = 3 for the control, T0, and T1 groups; *n* = 4 for the T2 group. ^##^*p* < 0.01 vs. the T0 group.

**Figure 6:** Cilengitide attenuates the apoptosis of abdominal aorta. (a) The representative image for TUNEL staining. Scale bar, 100 *μ*m. (b) Quantitative results of TUNEL-positive cells. *n* = 3 for the control, T0, and T1 groups; *n* = 4 for the T2 group. ^∗∗^*p* < 0.01 vs. the control group; ^#^*p* < 0.05 vs. the T0 group; ^##^*p* < 0.01 vs. the T0 group.

**Figure 7:** Cilengitide inhibits the VEGF expression in rabbit abdominal aortic plaque. (a, b) The representative image and quantification of VEGF-A in the plaque of the abdominal aorta. (c) The mRNA expression of VEGF in the plaque of the abdominal aorta. (d, e) The content of VEGF-A and VEGF-R2 was evaluated by ELISA in the plaque of the abdominal aorta. (f–h) Relative mRNA of *α*_v_, *β*_3_, and *β*_5_ in the plaque of the abdominal aorta. (i–l) The representative image and quantification of MMP-2, MMP-9, and MCP-1 expression in the plaque of the abdominal aorta. *n* = 3 for the control, T0, and T1 groups; *n* = 4 for the T2 group. ^∗∗^*p* < 0.01 vs. the control group; ^#^*p* < 0.05 vs. the T0 group; ^##^*p* < 0.01 vs. the T0 group.

**Figure 8:** The effect of cilengitide on the proliferation, migration, apoptosis, and tube formation of HUVECs. (a) The quantification of cell proliferation was evaluated by CCK-8 assay for HUVECs under treatment with different concentrations of cilengitide (0-10 *μ*M) for 24 hours. (b, c) The representative image and quantification of cell migration evaluation of HUVECs under treatment with different concentrations of cilengitide (0-10 *μ*M) for 24 hours. Scale bar, 100 *μ*m. (d, e) The representative image and quantification of apoptosis were evaluated by flow cytometry analysis for HUVECs under treatment with different concentrations of cilengitide (0-10 *μ*M) for 24 hours. (f) The representative image of tube formation assay of HUVECs under treatment with different concentrations of cilengitide (0-10 *μ*M) for 8 hours. (g–i) Quantification of the length of tubes, tube area, and the number of capillary-like structures for the tube formation assay of HUVECs. *n* = 5 for each group. Scale bar, 100 *μ*m. ^∗^*p* < 0.05 vs. 0 *μ*M; ^∗∗^*p* < 0.01 vs. 0 *μ*M.

**Figure 9:** Cilengitide treatment inhibits the mRNA expression of VEGF, *α*_v_, *β*_3_, and *β*_5_ of HUVECs. (a) Cilengitide inhibits the mRNA expression of VEGF under doses of 10 *μ*M. (b) Cilengitide did not affect the mRNA expression of *α*_v_. (c) Cilengitide inhibits the mRNA expression of *β*_3_ under doses of 10 *μ*M. (d) Cilengitide inhibits the mRNA expression of *β*_5_ under the doses of 0.1 *μ*M, 1 *μ*M, and 10 *μ*M. *n* = 5 for each group. ^∗^*p* < 0.05 vs. 0 *μ*M; ^∗∗^*p* < 0.01 vs. 0 *μ*M.

**Figure 10:** Cilengitide treatment inhibits the expression of VEGF and its downstream Ras/ERK/AKT signaling pathway of HUVECs. (a) Representative image of western blots for the protein expression of VEGF, Ras, p-ERK/EKR, and p-AKT/AKT under treatment with 0 *μ*M, 1 *μ*M, and 10 *μ*M cilengitide. (b–e) Quantification of the protein expression levels. *n* = 5 for each group. ^∗^*p* < 0.05 vs. 0 *μ*M; ^∗∗^*p* < 0.01 vs. 0 *μ*M.

**Figure 11:** Schematic illustration of the effect of cilengitide on the HUVECs. Recognizing the ligands with conserved arginine-glycine-aspartic acid (RGD) motifs, integrin *α*_v_*β*_3_ mediates the various activities of cell adhesion. Cilengitide has a high affinity for integrin *α*_v_*β*_3_ and inhibits relevant intracellular signaling. It inhibits the proliferation, migration, and tube formation of HUVECs but not affects apoptosis.

**Table 1:** List of primer sequence of target gene used in RT-qPCR.

Genes	Primers (F: forward, R: reverse)
VEGF-rabbit	F-5′-GGAGTACCCTGATGAGATCG-3′
	R-5′-CACATTTGTTGTGCTGTAGG-3′
*α*_V_-rabbit	F-5′-GGGTAGCGGGGAAGCAAG-3′
	R-5′-ACAGCTACGGAATAGCCCAA-3′
*β*_3_-rabbit	F-5′-GGAAAGATTGGCTGGAGGAA-3′
	R-5′-GGCATACCCCACACTCAAAG-3′
*β*_5_-rabbit	F-5′-TGCTCCAGAGAGGACTTCGG-3′
	R-5′-CGGATTGGTCTGGTACCTCG-3′
*β*-Actin-rabbit	F-5′-TGGACATCCGCAAGGACCTG-3′
	R-5′-GCTGGAAGGTGGAGAGCGAG-3′
VEGF-human	F-5′-AGGGCAGAATCATCACGAAGT-3′
	R-5′-AGGGTCTC GATTGGATGGCA-3′
*α*_V_-human	F-5′-AGCTGAGCTCATCGTTTCCATTC-3′
	R-5′-CCTTCATTGGGTTTCCAAGGTC-3′
*β*_3_-human	F-5*'*-GAGGTCATCCCTGCCTCAA-3′
	R-5′-CTGGCAGGCACAGTC ACAATC-3′
*β*_5_-human	F-5′-GGAGCCAGAGTGTGGAAACA-3′
	R-5′-GAAACTTTGCAAACTCCCTC-3′
GAPDH-human	F-5′-GGAGCGAGATCCCTCCAAAAT-3′
	R-5′-GGCTGTTGTCATACTTCTCATGG-3′

**Table 2:** Comparison of basic parameters of abdominal aorta in the three groups.

		Number of animals	Weight (kg)	Inner diameter (mm)	IMT (mm)	Heart rate (beats/min)	PSV (cm/s)	RI	VRI
Pretreatment	T0 group	3	2.917 ± 0.161	3.007 ± 0.198	0.300 ± 0.061	272.33 ± 26.86	105.37 ± 13.76	0.753 ± 0.049	1.030 ± 0.025
	T1 group	3	2.750 ± 0.050	3.393 ± 0.297	0.353 ± 0.045	287.67 ± 42.00	82.93 ± 10.88	0.733 ± 0.041	1.050 ± 0.061
	T2 group	4	2.807 ± 0.189	3.353 ± 0.284	0.330 ± 0.026	273.00 ± 15.49	111.30 ± 31.80	0.740 ± 0.014	1.017 ± 0.049
Posttreatment	T0 group	3	2.900 ± 0.166	3.220 ± 0.167	0.317 ± 0.081	238.33 ± 29.84	109.87 ± 30.80	0.713 ± 0.090	0.990 ± 0.078
	T1 group	3	2.683 ± 0.029	3.453 ± 0.256	0.340 ± 0.062	277.00 ± 24.25	89.30 ± 14.84	0.730 ± 0.050	1.003 ± 0.006
	T2 group	4	2.700 ± 0.214	3.148 ± 0.367	0.370 ± 0.014	262.75 ± 27.02	113.50 ± 17.33	0.755 ± 0.034	1.002 ± 0.040

Data are presented as means ± SEM. *p* value > 0.05 for all comparisons. IMT: intima-media thickness of abdominal aorta; PSV: peak systolic velocity; RI: resistance index; VRI: vascular remodeling index.

**Table 3:** Baseline characteristics of abdominal aortic plaque size and eccentricity index (EI) before cilengitide treatment in the three groups.

	Number of plaques	CGG (point)	Plaque size and EI detected by CUS			Plaque size and EI detected by CEUS		
			LD (mm)	AD (mm)	EI	LD (mm)	AD (mm)	EI
T0 group	3	3.667 ± 0.577	4.177 ± 0.289	0.620 ± 0.053	0.522 ± 0.085	3.833 ± 0.576	0.587 ± 0.023	0.487 ± 0.116
T1 group	5	3.400 ± 0.548	3.816 ± 1.269	0.588 ± 0.059	0.392 ± 0.102	3.722 ± 0.952	0.556 ± 0.043	0.408 ± 0.076
T2 group	7	4.571 ± 1.718	3.676 ± 1.006	0.663 ± 0.194	0.486 ± 0.116	5.027 ± 1.694	0.726 ± 0.184	0.533 ± 0.111

Data are presented as means ± SEM. *p* value > 0.05 for all comparisons. CGG: contrast agent grayscale (replace the grayscale with the number of the microbubbles shown in a plaque); LD: longitudinal diameter; AD: anteroposterior diameter; EI: eccentricity index; CUS: conventional ultrasound; CEUS: contrast-enhanced ultrasound.

**Table 4:** Comparison of changes in the degrees of aortic plaque size and eccentricity index (EI) after cilengitide treatment in the three groups.

	Number of plaques	CGG (point)	Changes in plaque size and EI detected by CUS			Changes in plaque size and EI detected by CEUS		
			LD (mm)	AD (mm)	EI	LD (mm)	AD (mm)	EI
T0 group	3	0.000 ± 1.000	−0.497 ± 0.571	−0.033 ± 0.083	−0.060 ± 0.059	0.408 ± 0.893	0.183 ± 0.163	0.104 ± 0.119
T1 group	5	1.000 ± 0.707	−0.488 ± 1.213	−0.058 ± 0.048	−0.018 ± 0.154	−0.396 ± 0.466	−0.024 ± 0.050^#^	−0.070 ± 0.086^#^
T2 group	7	1.571 ± 0.534^∗^	−0.624 ± 0.686	−0.079 ± 0.136	−0.131 ± 0.078	−1.603 ± 1.191^∗^	−0.104 ± 0.065^∗∗&^	−0.171 ± 0.072^∗∗&^

Data are presented as means ± SEM. ^#^T1 group compared with T0 group; ^∗^T2 group compared with T0 group; ^&^T2 group compared with T1 group; ^∗,#,&^*p* < 0.05, ^∗∗^*p* < 0.01. CGG: contrast agent grayscale (replace the grayscale with the number of the microbubbles shown in a plaque); LD: longitudinal diameter; AD: anteroposterior diameter; EI: eccentricity index; CUS: conventional ultrasound; CEUS: contrast-enhanced ultrasound. Plaques in the same site were measured for changes in LD, AD, and EI before and after treatment; Negative and positive values for LD and AD indicate that the plaques became smaller or larger after treatment, respectively; Negative and positive values for the EI reflected an increase or decrease of the lumen of the blood vessel.

## Data Availability

The data used to support the findings of this study are available from the corresponding author upon request.
